# Genetic Algorithm in Multimedia Dynamic Prediction of Groundwater in Open-Pit Mine

**DOI:** 10.1155/2022/8556103

**Published:** 2022-05-27

**Authors:** Runting Zhang, Shuzhao Chen, Zhouai Zhang, Wencheng Zhu

**Affiliations:** ^1^Production Technology Department, National Energy Baorixile Energy Co., Ltd., Hulun Buir 021000, Inner Mongolia Autonomous Region, China; ^2^School of Mines, China University of Mining and Technology, Xuzhou 221116, Jiangsu, China

## Abstract

This study is aiming at the nonlinear mapping relationship between the groundwater level and its influencing factors. Through the design and calculation process of matlab7 platform, taking the monitoring wells distributed in an open-pit mining area as an example, the short-term prediction of groundwater dynamics in the study area is carried out by using BP neural network model and BP neural network model based on genetic algorithm. Root mean squared error (RMSE), Mean absolute percent-age error (MAPE) and Nash–Sutcliffe efficiency (NSE) are used coefficients,, and the results were compared with BP neural network and stepwise regression model. From the results of the comparative analysis, the genetic algorithm optimized the BP neural network model in the training phase and the test phase, the RMSE was 0.25 and 0.36, the MAPE was 6.7 and 8.13%, and the NSE was 0.87 and 0.72, respectively. The BP neural network model optimized by genetic algorithm is obviously superior to the BP neural network model, which is an ideal prediction model for short-term groundwater level. This model can provide a prediction method for groundwater dynamic prediction and has a good application prospect.

## 1. Introduction

The change of groundwater level is a very complex natural process, and it is the comprehensive effect of groundwater system stimulated by multiple inputs [1]. Factors such as precipitation, evaporation, and artificial mining can be regarded as inputs to the system, and the groundwater level can be regarded as the output of the system [2]. At the same time, due to the spatial variation of the aqueous system, there will be data variability in the actual research process, and some precise research methods often fall into a variety of dilemmas when describing the nonlinear relationship of groundwater systems [3]. Numerical methods can describe irregularly shaped regions and aquifers with heterogeneity, anisotropy, and complex boundary conditions, can deal with river infiltration, atmospheric precipitation replenishment, changes in the temporal and spatial distribution of various pumping, drainage and evaporation, so as to solve complex problems that are not easy to solve by other calculation methods; however, the numerical method as a distributed parameter model has high requirements on the quantity and accuracy of the data [4]. The degree of research in some areas cannot meet the calculation requirements of the distributed parameter model, and it is more suitable from a system point of view, treat them as a whole, apply system theory to establish a centralized parameter model, analyze, study, and solve problems as a whole [5]. In recent years, the neural network method due to its powerful ability to deal with nonlinear dynamic systems, and it has been widely used and promoted in groundwater dynamic prediction [6]. In response to this research question, Supreetha et al.. elaborated on the advantages of artificial neural network models compared with traditional simulation models [7]. Mohammadrezapour and Kisi used neural network models to select precipitation, evaporation, surface runoff, and other information related to shallow groundwater dynamics and used them to predict phreatic groundwater dynamics [8]. Xia et al. successfully predicted the groundwater dynamics of semiconfined aquifers using the neural network method based on extraction volume and hydrometeorological factors [9]. On the basis of the current research, through the design and calculation process of MATLAB 7 platform, taking the monitoring wells distributed in an open-pit mining area as an example, the short-term prediction of groundwater dynamics in the study area is carried out by using BP neural network model and BP neural network model based on genetic algorithm. Root mean squared error (RMSE), Mean absolute percent-age error (MAPE) and Nash–Sutcliffe efficiency (NSE) are used as coefficient, and the results were compared with BP neural network and stepwise regression model. According to the results of comparative analysis, RMSE of BP neural network model optimized by genetic algorithm were 0.25 and 0.36, MAPE were 6.7 and 8.13%, AND NSE were 0.87 and 0.72, respectively, in the training stage and test stage. The BP neural network model optimized by genetic algorithm is obviously superior to the BP neural network model, which is an ideal prediction model for short-term groundwater level.

## 2. Method

### 2.1. Based on GA-BP Neural Network Model

#### 2.1.1. BP Neural Network

Back-propagation (BP) neutral network was studied and designed by RUMELHART, MCCELLAND and their research group in 1986. It is a multi-layer forward neural network composed of input layer, hidden layer, and output layer. Nodes from the front layer to the back layer are connected by network weights, and there is no coupling in nodes of the same layer. Activation functions of input layer and hidden layer are usually Sigmoid type, as shown in the following formula:

(1) $$\begin{array}{c} f\left(x\right)=\frac{1}{1+e^{-x}}. \end{array}$$

The learning and training process of BP neural network is divided into two parts, and they are the forward propagation network input signal and the backward propagation error signal, trained according to the way of having a tutor. In the process of forward propagation, the input factor is passed from the input layer to the output layer through the hidden layer calculation layer by layer, each neuron in the output layer outputs the network response corresponding to the input mode, If the output layer cannot get the expected output factor, at this time, the error is transferred to the back propagation, according to the principle of reducing the error between the expected output and the actual output, from the output layer back to the middle layers, and finally back to the input layer, and modify the weights and ratings of each connection layer by layer. As this error back propagation training continues, the correct rate of network response to input patterns has also been continuously improved, and so on, until the output error reaches the allowable range or the number of training times reaches the predesigned number of times [10].

#### 2.1.2. GA-BP Neural Network Model

In the application of BP neural network example, most models adopt the form of error back propagation; however, the BP neural network model will have local minima and overfitting in the training and prediction process, and it can only be carried out according to the set parameters, and it is impossible to search for the optimal solution for the weights and thresholds of the hidden layer [11]. The basic idea of GA-BP neural network is to find the most suitable network connection weight and network structure by taking advantage of the global search characteristic of genetic algorithm and changing the way that BP algorithm adjusts the weight of neural network depending on the guidance of gradient information. The algorithm has the global search technology of adaptive probability, breaks through the traditional rule search method, makes the search process more flexible, and simultaneously in the multipeak problem has the ability to grasp the overall situation.

#### 2.1.3. Stepwise Regression

The stepwise regression model first considers the degree of influence of each variable on the dependent variable, introduces the significance of the independent variables into the equation in order from strong to weak, and the less significant ones will not be introduced. But in the process of introducing variables, independent variables with higher significance in the original equation may lose significance due to the introduction of new variables and be discarded. In this way, the culling is continuously looped, until the independent variables in the regression equation are all significant to the dependent variable, and at the end of the loop, the optimal regression equation is obtained. The steps of stepwise regression are as follows [12].

Set up multiple linear regression equations, establish multiple linear regression equations, and use the least square method to calculate the undetermined coefficients of the linear regression equation as shown in the formula:

(2) $$\begin{array}{c} s_{e}=\sqrt{\frac{\sum_{i=1}^{n}{\left(y_{i}-{\hat{y}}_{i}\right)}^{2}}{n-m-1}},\\ s_{bi}=\frac{s_{e}}{\sum_{i=1}^{n}{\left(x_{1}-\bar{x}\right)}^{2}}. \end{array}$$

In the formula, *s*_*e*_ is the standard estimation error; *s*_*bi*_ is the standard deviation of *b*_*i*_; *b*_*i*_ is the regression coefficient; *y*_*i*_ is the original value of the dependent variable; ${\hat{y}}_{i}$ is the predicted value of the dependent variable; *x*_*i*_ is the independent variable; $\bar{x}$ is the average value of the independent variable; *n* is the number of samples; *m* is the number of constraint conditions, and the test value is calculated.

(3) $$\begin{array}{c} t_{i}=\left|\frac{b_{i}}{s_{bi}}\right|. \end{array}$$

In the formula, *t*_*i*_ is the test value of *x*_*i*_.

Through the significance level *α* and the degree of freedom *f*, check the two-sided percentile table of the *t* distribution to find the critical value *t*_*a*_. The formula is as follows:

(4) $$\begin{array}{c} f=n-m-1. \end{array}$$

In the formula, *f* is the degree of freedom.

If the independent variable *t* test |*t*_*i*_|_min_ < *t*_*a*_, then this variable is not significant, after removing this variable, return to formula (2) loop calculation, until |*t*_*i*_|_min_ ≥ *t*_*a*_, it shows that all independent variables have high significance to the dependent variable.

The stepwise regression is over, and the optimal regression model is obtained as follows:

(5) $$\begin{array}{c} y_{i}=a_{0}+a_{1}x_{1}+a_{2}x_{2}+...+a_{i-m}x_{i-m}. \end{array}$$

In the formula, *y*_*i*_ is the groundwater dynamic prediction at time *i*; *x*_1_, ..., *x*_*i*_ is the value of the input variable from 1 to I, and *a*_*i*_, ..., *a*_*i*−1_ is the undetermined coefficient.

#### 2.1.4. Evaluation Index of the Model

In order to better evaluate the prediction effect of the established model, the following indicators are used to evaluate the model.

*Overall Prediction Accuracy*. The validity and capability of the model were predicted accurately, and the prediction accuracy was expressed by RMSE:

(6) $$\begin{array}{c} \text{RMSE}=\sqrt{\frac{\sum_{i=1}^{n}{\left(y_{i}-{\hat{y}}_{i}\right)}^{2}}{n}}. \end{array}$$

In formula (6), *y*_*i*_ is the measured value; ${\hat{y}}_{i}$ is the predicted value; and *n* is the number of samples.

Mean absolute error. MAPE calculates the relative error variable between the predicted value and the actual value through comparison term by term. Therefore, MAPE is an unbiased statistic, and the prediction ability of the model can be seen as follows:

(7) $$\begin{array}{c} \text{MAPE}=\frac{1}{n}\sum_{i=1}^{n}\left|\frac{{\hat{y}}_{i}-y_{i}}{y_{i}}\right|\times 100\%. \end{array}$$

Nash efficiency coefficient (NSE ey coefficient) model is used to evaluate the predictive power of hydrological models, and it can describe the tracking ability of the predicted value to the measured value, and the calculation method is as follows:

(8) $$\begin{array}{c} \text{NSE}=1-\frac{\sum_{i=1}^{n}{\left(y_{i}-{\hat{y}}_{i}\right)}^{2}}{\sum_{i=1}^{n}{\left(y_{i}-\bar{y}\right)}^{2}}, \end{array}$$

where $\bar{y}$ is the average value of measured values and the value range of NSE is (−*∞*, 1]. When the calculated value is close to 1, the stability of prediction is higher. When the value of NSE is close to 0, the predicted results are closer to the mean value of the measured samples. When the value of NSE is less than 0, it indicates that the model prediction results are unreliable.

### 2.2. Selection and Preprocessing of Input Variables

#### 2.2.1. Selection of Input Variables

A certain county is located in the west of the Huaibei Plain, with flat and open terrain, the groundwater type is a single loose rock pore water. According to the relationship between groundwater burial conditions, hydraulic characteristics, atmospheric precipitation, and surface water, groundwater is divided into shallow groundwater and deep groundwater from top to bottom. The data of a county from 1974 to 1999 is used to train the model, and the data from 2000 to 2010 is used to test the model [13]. The selection of model input samples has an important influence on the calculation results of the model, precipitation is the main source of groundwater, and the previous groundwater has a strong correlation with the groundwater of the month, the groundwater 3 months, 4 months, 5 months, 6 months, and 7 months before the forecast period are used as input samples in the GA-BP neural network. The accuracy of fitting and forecasting groundwater as the input sample in the first 5 months of the period to be predicted in a certain county is the highest; therefore, the rainfall in the month before the forecast period in a certain county and the groundwater in the first 5 months are selected as input samples, as listed in Table 1 [14].

#### 2.2.2. Pretreatment

Due to the different dimensions of the selected input samples, it cannot be directly used as an input sample; therefore, it must be normalized. Its purpose is mainly to accelerate the convergence speed of the neural network, eliminate errors caused by different dimensions, and use linear function conversion to process the original data, the specific processing methods are as follows:

(9) $$\begin{array}{c} y=\frac{\left(x-x_{\min}\right)}{\left(x_{\max}-x_{\min}\right)}. \end{array}$$

In formula (9), *x* and *y* are the original input data and preprocessed data, respectively; *x*_max_ and *x*_min_ are the maximum and minimum values of the original data, respectively.

## 3. Results and Analysis

### 3.1. Model Establishment and Training

Use MATLAB R2014a to write a program to establish a GA-BP neural network model for a county in Anhui Province.

For groundwater simulation and prediction, divide the data into training samples and test samples, and in order to make the model have a higher fitting accuracy, use monthly data from 1974 to 1999 for training samples. At the same time, the monthly data of a certain county from 2000 to 2010 is used for the inspection sample, and establish GA-BP neural network model. The nodes in the input layer of the model consist of rainfall during the period to be predicted (1-1), and the groundwater (*t* − 1) composition for the first 5 months to be predicted, and the output layer node of the groundwater in a certain county during the period to be predicted. The number of nodes in the hidden layer of the neural network has a great impact on the neural network, if the number of nodes is small, the network performance may be extremely poor, if the number of nodes is too much, the training is easy to fall into the local minimum [15]. In order to avoid the blindness of selection, on the basis of BP neural network, write the loop code for the number of hidden layer nodes. according to experience, the initial value of the number of nodes in the hidden layer is 15, the number of termination nodes is 40. When the number of nodes in the hidden layer is 19, the relative average error of the model training and prediction phase is the smallest. The relative average error of nodes in the hidden layer of the GA-BP neural network model from 15–40 training and prediction stages is shown in Figure 1. The structure of BP neural network is 7 : 19 : 1. Set the population number to 10 during the evolution of the genetic algorithm, the evolutionary algebra is 20, the mutation probability is 0.1, and the crossover probability is 0.1. According to the above GA-BP neural network model, the weights and thresholds between the layers of the BP neural network optimized by the genetic algorithm can be obtained [16].

### 3.2. Model Test

After the GA-BP neural network model is established, its accuracy needs to be tested. In order to test the effect of the GA-BP neural network model, compare the model with the stepwise regression model 4 and the BP neural network model, perform groundwater fitting and prediction during the period to be predicted [17]. Stepwise regression will gradually eliminate the factors of the GA-BP input layer, the ranking of the contribution of the correlation is as follows: groundwater in the period to be predicted (*t* − 2) > rainfall in the period to be predicted in a county (*t* − 1) > groundwater in a certain county during the time to be predicted (*t* − 1) > groundwater in a certain county during the time to be predicted (*t* − 3) > the groundwater during the period to be predicted in a county (*t* − 1) > the groundwater during the period to be predicted in county A (*t* − 4) > the groundwater in a certain county during the period to be predicted (*t* − 5), excluding the last two input samples, the first 5 input samples are retained [18]. The reason is that the rainfall (*t* − 1) and the previous (*t* − 1), (*t* − 2) and (*t* − 3) months of the area to be forecasted during the period of rainfall (*t* − 1) are close to the groundwater in the period to be predicted, the impact is strong. Early groundwater in County A reflects the development trend of groundwater levels in adjacent areas [19]. Use stepwise regression to select impact factors for simulation and prediction, and the final regression equation is shown in the following formula [20]:

(10) $$\begin{array}{c} y=0.6335-0.0016x_{1}+0.9629x_{2}-0.1856x_{3}+0.1118x_{4}-0.1319x_{7}. \end{array}$$

In formula (10), *x*_1_ is the rainfall during the period to be predicted in a certain county (*t* − 1); *x*_2_ is the groundwater (*t* − 1) during the period to be predicted in a county; *x*_3_ is the groundwater (*t* − 2) of a certain county during the period to be predicted; *x*_4_ is the groundwater in a certain county during the period to be predicted (*t* − 3); *x*_7_ and groundwater for the period to be predicted in Lixin County (1-1) [21].

The input variables of the BP neural network and the GA-BP neural network are the same, and the output results are compared [22]. Taking into account that the groundwater is too deep or too shallow will bring greater harm, separately for the 10% maximum (deepest) and 10% minimum (shallowest) samples of the long series of groundwater series—the above three indicators are used to evaluate the maximum and minimum groups predicted by the three models [23]. The process of predicting groundwater by the above three models is shown in Figure 2, and the evaluation indicators of each plan are listed in Table 2 [4].

From the analysis of Figure 2 and Table 1, it can be seen that, the GA-BP neural network has better results than the BP neural network and the stepwise regression model in the values of the indicators in the two stages. The accuracy of simulation and prediction is the highest among the three models. It shows that the GA-BP model fully combines the advantages of genetic algorithm and neural network, overcome the problems of local optima and poor convergence ability, and the prediction accuracy and fitting accuracy are close and high, which fully demonstrates the good generalization ability of the GA-BP model [24].

Based on the above analysis, the accuracy and stability of prediction from high to low are ga-BP model > BP neural network > stepwise regression. The RMSE of stepwise regression training and prediction stage was 0.71 m lower than that of BP neural network, MAPE of two stages was 8.15% and 3.13% higher than that of BP neural network, and NSE of neural network was 0.1 higher than that of stepwise regression. At the same time, the NSE of stepwise regression is less than 0 in the stability of maximum and minimum prediction, which fully shows that the stability of stepwise regression is not reliable in the stability of maximum and minimum prediction, and the BP neural network is superior to the stepwise regression model in the values of RMSE and MAPE of maximum and minimum prediction. The reason is that stepwise regression is based on linear theory to solve linear problems. However, due to the influence of hydrology, water use, artificial mining, and other factors, groundwater presents a complex nonlinear relationship, and stepwise regression cannot achieve good results in solving the nonlinear relationship, so the phenomenon of poor prediction accuracy appears in this paper. However, BP neural network mainly relies on these long-term observation data and has strong learning ability. When the input factors change and the complex nonlinear relationship is presented, it only needs to let the model learn again to track the changes of the system. Therefore, BP neural network model is superior to stepwise regression model in solving this problem.

## 4. Conclusion

BP neural network model and BP neural network model based on genetic algorithm, a short-term forecast of the groundwater dynamics in the study area was carried out. RMSE, MAPE, and NSE were used to compare the results with BP neural network and stepwise regression model. The combination of genetic algorithm and BP neural network not only gives full play to the generalization mapping ability of BP neural network and the global convergence ability of genetic algorithm but also overcomes the phenomenon that the local regulation ability of genetic algorithm is weak, which further improved the forecasting ability and stability.

## Figures and Tables

**Figure 1:** The average relative error of different nodes in the hidden layer of the GA-BP neural network model during the training and prediction stages.

**Figure 2:** Groundwater prediction process of a county from 2000 to 2010 based on three models.

**Table 1:** Relative errors of groundwater before different prediction periods by GA-BP neural network.

Project	Groundwater before the forecast period				
	The first 3 months	The first 4 months	The first 5 months	The first 6 months	The first 7 months
Training relative mean error	14.79	10.26	7.61	11.22	11.35
Relative mean error of prediction	18.52	14.21	9.22	14.52	17.82

**Table 2:** Model simulation and prediction performance parameter analysis and comparison.

Model	RMSE				MAPE				NSE			
	Predict	Train	Max	Minimum	Predict	Train	Max	Minimum	Predict	Train	Max	Minimum
Genetic algorithm optimization, that is, BP neural network returns home	0.33	0.21	0.31	0.10	9.20	7.61	8.61	9.60	0.84	0.91	0.62	0.39
	0.41	0.26	0.34	0.41	13.42	10.39	12.69	19.59	0.83	0.81	0.51	0.35
	0.47	0.34	0.48	0.52	21.39	13.49	10.61	32.65	0.71	0.76	−0.95	−0.93

## Data Availability

The data used to support the findings of this study are available from the corresponding author upon request.
